RETRACTED

# Research on Segmentation of Brain Tumor in MRI Image Based on Convolutional Neural Network

**DOI:** 10.1155/2022/7911801

**Published:** 2022-08-05

**Authors:** Yurong Feng, Jiao Li, Xi Zhang

**Affiliations:** ^1^Department of Radiology, The First People's Hospital of Jingmen City, Hubei, China; ^2^Neurosurgery, The First People's Hospital of Jingmen City, Hubei, China

## Abstract

Brain tumors are the brain diseases with the highest mortality and prevalence, and magnetic resonance imaging has high-resolution and multiparameter. As the basis for realizing the quantitative analysis of brain tumors, automatic segmentation plays a vital role in diagnosis and treatment. A new network model is proposed to improve the accuracy of convolutional neural network segmentation of brain tumor regions and control the parameter space scale of the network model. The model first uses a convolutional layer composed of a series of 3D convolution filters to construct a backbone network for feature learning of input 3D MRI image blocks. Then, a pyramid structure constructed by a 3D convolutional layer is designed to extract and fuse features of tumor lesions and context information of different scales and then classify the fused feature at the voxel level to obtain segmentation results. Finally, a conditional random field is used to postprocess segmentation results for structured refinement. By designing massive ablation experiments to analyze the sensitivity of the essential modules of the comparison network, the results confirm that our method can better solve the problems faced by the traditional fully connected convolutional neural network.

## 1. Introduction

Brain tumors are very harmful to the human body. Brain tumors are divided into two types: the first is called primary brain tumors, and the other is called secondary brain tumor. This tumor originates from a malignant tumor outside the brain, starts in other parts of the body, and then spreads to the brain. Computed tomography (CT), magnetic resonance imaging (MRI), and ultrasound are imaging techniques commonly used in medical anatomy. Among them, because MRI can image human brain soft tissues and brain tumors more clearly than CT, MRI's specific imaging features are as follows: (1) noninvasive imaging. Magnetic resonance imaging is related to nuclear magnetic resonance, which uses electromagnetic waves and does not cause ionizing radiation damage to the human body, so it is called magnetic resonance imaging. (2) Multiparameter imaging. MRI parameters mainly include T1, T2, and proton density, which can provide more clinical diagnostic information, unlike CT, which has only one absorption coefficient parameter. (3) High-contrast imaging. Hydrogen protons are the most abundant atomic nuclei in the human body. They are distributed anywhere in the body. Depending on the strength of the magnetic resonance signal of hydrogen protons in different tissues, high-contrast imaging of tissues can be achieved. (4) Multidirectional imaging. MRI only needs one scan to get a three-dimensional image. It is easy to view slice images in any direction, such as coronal plane, sagittal plane, and cross-section. (5) No bone artifact interference. When using X-ray, CT, and ultrasound diagnostic equipment to check, due to the overlap of bones and gas, the resulting images usually have artifacts that interfere with the diagnosis. However, MRI has no such interference [1–5].

RETRACTED

MRI plays a vital role in brain tumor detection and treatment. Accurately drawing the boundary contour of the visible exudate of the tumor can effectively help quantify the size of the lesion and the cumulative rate of its longitudinal data. However, the shape of complex high-grade tumors of the recorded heterogeneous media can be obtained. However, tumor segmentation that includes all intact parts becomes more challenging due to their high proliferation, growth rate, and variability in appearance. Manual segmentation is subject to the observer's own influence, making automatic segmentation more demanding.

Generally, the treatment plan for patients with brain tumors varies according to the histopathological type and the location of the disease. Before and after treatment, it is necessary to carry out some measurements and analysis that are helpful for doctors to diagnose, formulate, and modify the patient's treatment plan or program. For example, the quantitative analysis of brain tumors refers to the measurement of the maximum diameter, volume, and the number of brain lesions to quantify the response before and after treatment of brain tumors. However, reliable measurement depends on accurate segmentation. However, the segmentation processing of brain tumor imaging depends more on the experience of anatomy experts. This processing is not only time-consuming and laborious, but the results obtained are subjective. Different people or the same person usually draws different conclusions at different times [6–10].

Therefore, the best way to solve the above problems is to design an automatic segmentation algorithm, which is also one of the development directions of segmentation technology. However, brain tumors can appear anywhere, and the size and shape are also ever-changing, with different patients having considerable differences. MRI images are affected by degraded conditions such as noise and local volume effects, causing uneven grayscale of the image. There may be similar grayscale values between the tumor and normal tissues and subregions within the tumor. These characteristics and uncertainties bring great difficulties to the reliability of brain tumor segmentation algorithms and the accuracy of results. Therefore, the study of new methods and new ideas for MRI image brain tumor segmentation is extremely important. This requires researchers to invest more energy in image segmentation as well as look forward to finding new methods to solve practical problems.

RETRACTED

As a kind of artificial neural network, CNN can actively learn features. And within a certain range, as the number of layers increases, the more abstract the learned features, the better the segmentation effect. It has become a research hotspot in the field of image recognition. Havaei e al. [11] divide the training process for the network into two stages and extract the local and overall features of the image at the same time. This method has made great progress in the segmentation effect. However, some patients have very low accuracy on the enhancing indicators in the core and complete areas. The main reason is that the boundary between the enhanced and nonenhanced areas is unclear, and this model autonomously learns the features in the original image. Compared with traditional convolutional neural networks that only operate on one scale, Zhao and Jia [12] convolve images on different scales. However, because there is no image preprocessing before training, the variance obtained in the experiment is large, and the experimental results are not ideal. Most methods will choose to use 2D filters for feature extraction, but using 3D filters can make fuller use of image features. Wang et al. [13] proposed joint training of deep and shallow networks based on end-to-end networks and achieved better performance. Zhao et al. [14] use the output of a cascaded network as an additional input for the next network. The success of convolutional neural networks was mainly attributed to the following points: the effective use of GPU accelerates the training speed of the network. The activation functions such as ReLU and regularization methods such as dropout have improved the accuracy of the network; a large amount of training data can be used for model training.

Pereira et al. [4] used a shallow model for classification. The model has two convolutional layers, and the maximum pooling step of the convolutional layer is 3. There is also a fully connected layer and a Softmax layer. Hussain et al. [15] evaluated the usefulness of a 3D filter, although most authors chose 2D filters. The 3D filter benefits the 3D characteristics of the image, but it increases the computational burden. Some proposals have evaluated a two-path network, allowing one branch to receive larger blocks than the other and therefore have a larger contextual view of the image [11]. Lyksborg et al. [16] used a binary CNN to identify intact tumors, and then, before multiclass CNNs identify the subregions of tumors, cellular automata were used to smooth segmentation. Rao et al. [17] extract blocks on each voxel plane, train CNN in the MRI sequence, concatenate the FC layer output with each CNN regression, and use it to train the RF classifier. Dvorák and Menze [18] divided the brain tumor region segmentation task into binary subtasks and proposed structured prediction using CNN as a learning method. The blocks in the tag are all gathered into the dictionary of tag blocks, and the CNN must be able to predict the membership of each cluster input. Simonyan and Zisserman [19] proposed using a smaller 3 × 3 kernel operator to obtain a deeper structure of CNNs. Some other experimental research works about brain tumors were studied by different scholars, which were given in [20–24]. With smaller kernel operators, we can extract more convolutional layers, which have the same ability to accept larger kernel operators. For example, two concatenated convolutional layers have the same effective acceptance but will have a smaller weight value. At the same time, they also have certain advantages.

RETRACTED

## 2. Method

The model proposed in our work includes the following aspects: 3D atrous convolutional neural network, multiple feature learning, and conditional random field. The whole frame structure is illustrated in Figure 1.

### 2.1. Dataset and Evaluation Metric

This experiment uses clinical imaging data obtained from the BraTS 2013 dataset provided by MICCAI (Table 1). BraTS 2013 provided MRI imaging information of 65 patients with glioma, including 51 patients with high-grade glioma (HGG) and 14 patients with low-grade glioma (LGG). The MRI image of each patient has the same direction and four imaging modalities. For ease of description, this article refers to the two data sets of Challenge and LeaderBoard as the BraTS 2013 test set.

The BraTS data set evaluates the performance of the algorithm by calculating indicators under the three categories of intact tumor (WT), tumor core (TC), and enhanced tumor core (EC). Specific indicators include DICE similarity coefficient (DSC). The experimental environment is shown in Table 2.

### 2.2. 3D Atrous Convolutional Network

In an ordinary full convolutional network, due to repeated pooling and convolution sliding calculations, the resolution of the feature map will decrease layer by layer. Although in the classification task, this method will get a highly abstract and dimensionally reduced feature matrix, but for the fine semantic segmentation task, it will also lead to the loss of some important spatial information. To overcome this shortcoming, an atrous convolution filter that replaces the pooling layer in ordinary DCNNs is proposed to eliminate the downsampling operator so that the network can generate denser semantic feature maps for segmentation tasks. This chapter expands the original atrous convolution filter used for semantic segmentation of 2D images into a 3D atrous convolution filter. Simply understand, atrous convolution filter is realized by jacking between the weights inside the filter core of the ordinary nonzero convolution filter. It was proposed to calculate undecimated wavelet transform effectively. By inserting atrous, a larger receptive field can be obtained.

RETRACTED

Taking the one-dimensional input signal *x*[*i*] as an example, the output *y*[*i*] calculated by the atrous convolution is as

(1) $$\begin{array}{c} y\left[i\right]=\overset{K}{\underset{K=1}{\sum }}x\left[i+r\times k\right]w\left[k\right]. \end{array}$$

*r* is the sliding or sampling step of the filter in the corresponding input signal. When the filling number is close to the atrous rate, the network is able to learn denser features. By changing the atrous rate, the density of feature learned by the atrous convolutional neural network can be controlled.

In addition, by modifying the atrous rate and stride, the atrous convolution filter can increase the receptive field. Suppose there is a 3D ordinary convolution filter *k*^*x*,*y*,*z*^ of size *k* × *k* × *k*, and (*x*, *y*, *z*) represents the axial, sagittal, and coronal positions of the MRI image. Then, the size of the convolution kernel of atrous convolution filter with atrous rate is calculated as follows:

(2) $$\begin{array}{c} k_{\text{new}}^{x,y,z}=k^{x,y,z}+\left(k^{x,y,z}-1\right)\times \left(r-1\right). \end{array}$$

This formula is equivalent to not changing the original input signal and sampling the ordinary convolution filter by adding *r* − 1 zeros between the filter weights. Therefore, if the receptive field size of the *l* − 1 network layer is RF, the receptive field size of the *l*th 3D convolutional network layer can be calculated by the following formula:

(3) $$\begin{array}{c} {RF}_{l}^{x,y,z}={RF}_{l-1}^{x,y,x}+\left[k^{x,y,\text{z}}+\left(k^{x,y,z}-1\right)\times \left(r-1\right)\right]\times S_{l}^{x,y,z}\\ S_{l}^{x,y,z}=\overset{l}{\underset{i+0}{\prod }}S_{i}^{x,y,z}. \end{array}$$

If a certain 3D image block is represented as *I*^*x*,*y*,*z*^, then the feature map size *O*^*x*,*y*,*z*^ output in the *l*th network layer is

(4) $$\begin{array}{c} O^{x,y,z}=\left[\frac{I^{x.y.z}+2P^{x,y,z}-{RF}_{l-a}^{x,y,z}}{S_{l}^{x,y,z}}+1\right]. \end{array}$$

The input size of this chapter is larger than the receptive field of the convolutional neural network. Using this strategy, the final Softmax layer will generate multiple predictions at the same time. As long as the receptive field of the network can cover all inputs without filling, all predictions are possible, avoiding repeated convolution operations on the same voxel, thereby reducing computational cost and memory load.

RETRACTED

Although the atrous convolution will increase the filter size, only a nonzero filter value can obtain a response, and the filter parameters and the amount of calculation remain unchanged. Therefore, atrous convolution provides the best trade-off between computation and dense prediction. In view of this, this chapter designs a stacked deep convolutional neural backbone network including 3D hollow convolutional layers for feature learning. As the receptive field increases, CNN can learn more multilevel features, integrating tumor tissue and surrounding context information to refine the tumor boundary better. Subsequent experimental results show that both of these features make the model obtain a significant improvement.

### 2.3. Multiscale Feature Learning

If the training data set contains samples of different scales, then CNN can use these samples to perform multiscale feature learning. This mechanism enables CNN to segment lesions of different sizes. Generally speaking, multiscale processing methods can be divided into two categories, namely, multi-input multifeature output and single-input multifeature fusion output.

The first method is easy to understand: to construct a pyramid formed by multiple scaled versions of the image for the input image and then input these scaled images one by one into parallel CNN branches that share the same parameters for multiscale feature extraction. Multichannel architecture can be regarded as this type of design style. This type of method uses dual-channel CNN and different input sizes for multiscale feature extraction and medical image segmentation. In order to obtain the final result, the feature maps output by each parallel branch will be upsampled to the original input size and then spliced before input to the final classification layer. Although this multiscale processing significantly improves the segmentation accuracy, each branch network needs to pass all the pictures in the pyramid one by one, and this calculation is quite redundant. Therefore, using this method should weigh the computational cost and accuracy of all scale data input to each branch. The second method uses the spatial hierarchy of the feature matrix constructed by CNN for segmentation. This design style considers the hierarchical feature maps of objects of different scales; that is, in the absence of image pyramids, only single-scale image input is available. This structure is also called a feature pyramid. Using this strategy, some methods in recent years first use a general CNN as an encoder to extract hierarchical features and then add additional modules as a decoder. For example, a deconvolution filter or interpolation method is used to reconstruct and merge the original resolution of the feature map. In addition, inspired by the spatial pyramid pooling technology, the resampling convolution filtering technology also enables objects of any scale to be accurately predicted. The hollow space pyramid pooling can effectively obtain multiscale information using this kind of resampling technology. The pooling technology is implemented using multiple parallel atrous convolutional layers with different atrous rates. Each parallel branch extracts different scale features through the fusion operation to produce the final result.

RETRACTED

This chapter uses the generated feature map to have this inherent multiscale feature and designs a 3D structure module to be added to the backbone. This module is named the hollow convolution feature pyramid. The feature map is input into each branch composed of 3D atrous convolutions. In addition, the proposed network inserts an upsampling layer between the hollow convolutional layer and the splicing layer of each branch to expand the feature map size of this layer to make it consistent with the previous branch, so as to achieve different levels of feature map splicing operations.

### 2.4. Postprocessing Method Based on Conditional Random Field

With the increase of the network layer, the probability map output by CNN becomes smooth with the increase of the receptive field and spatial context. Although CNN can predict the existence and rough location of the target through the probability map output by Softmax, some noises in the input and local minima during the optimizing process will be passed to the final output layer by the network. This will result in the loss of edge features, which will affect the segmentation effect. In order to solve this problem, this section expands the original fully connected CRF to 3D form as a postprocessing method, which can make the final segmentation result more structured.

For a 3D image *I* as input, the voxel set of this image is denoted as {*I*_*i*_|*i* = 1, ⋯, *M*}; its label set function is *Y*. Through fully connected CRF, the image segmentation issue can be transformed into an optimization issue and solved as follows:

(5) $$\begin{array}{c} E\left(Y\right)=\overset{M}{\underset{i=1}{\sum }}\Phi \left(y_{i}^{u}\right)+\underset{M}{\sum }\Psi \left(y_{i}^{u},{\text{y}}_{j}^{v}\right). \end{array}$$

The binary potential function Ψ uses the form of a fully connected graph to measure the cost of assigning labels *u* and *v* to voxel at the same time, that is,

(6) $$\begin{array}{c} \Psi \left(y_{i}^{u},y_{j}^{v}\right)=\mu \left(u,v\right)k\left(f_{i},f_{j}\right). \end{array}$$

If the cost function is defined as a linear combination of a set of Gaussian kernels, the model can use the mean-field approximation method for inference. Therefore, the expression can be further written as

(7) $$\begin{array}{c} \Psi \left(y_{i}^{u},y_{j}^{v}\right)=\mu \left(u,v\right)\overset{k}{\underset{m=1}{\sum }}w^{\left(m\right)}k^{\left(m\right)}\left(f_{i},f_{j}\right). \end{array}$$

RETRACTED

## 3. Results and Discussion

### 3.1. Comparison with Other Methods

This section uses the test set of BraTS 2013 to compare the proposed method with cutting-edge methods. The mainstream methods include Hammoude measure (HM) [20], multimodal magnetic resonance (MMR) [21], fully automatic (FA) [22], automatic brain tissue (ABT) [23], and stereotactic brachytherapy (SBT) [24]. The result is shown in Figure 2.

It can be observed that the method proposed in this paper obtains competitive results on the BraTS 2013 data set, and the proposed method has obvious advantages compared with cutting-edge methods on the task of complete tumor segmentation.

### 3.2. Evaluate the Effectiveness of Atrous Convolution

Figure 3 shows the average evaluation results of these backbone networks on various indicators, where StdNet represents a standard convolutional neural network with a pooling layer. All the atrous ratios are set to 2 for the convolutional layer with atrous instead of the pooling layer. AConvNet.2 means that the second layer of the backbone network is a hollow convolutional layer. By analogy, AConvNet.3 and AconvNet.4, respectively, indicate that the 3rd and 4th layers are hollow convolutional layers.

It can be observed that the segmentation effect obtained by the backbone network constructed by the hollow convolutional layer is better than the backbone network constructed by the standard convolutional layer and the pooling layer. The experimental results confirmed that using this single-step hollow convolutional layer instead of the pooling layer to expand the receptive field of the network can effectively prevent the information flow from losing information during the transmission process. In addition, the results of the evaluation and comparison also reflect that the third layer of the backbone network AConvNet.3 composed of atrous convolution achieves the best segmentation effect. Therefore, this chapter uses AConvNet.3 as the baseline model for subsequent experimental comparison and analysis.

RETRACTED

### 3.3. Evaluate the Impact of Input Size

In this section, we use slices of different sizes as input to train the corresponding baseline models and study their influence on the segmentation effect. The block sizes set in the experiment in this section are, respectively, 19 × 19 × 19, 25 × 25 × 25, and 37 × 37 × 37 (mm). Use the BraTS 2013 training set to train the network with the above parameter settings and evaluate the comparison on the test set.  Figure 4 shows the average value of each index compared.

It can be seen from the above comparison results that when the receptive field is 17 × 17 × 17, setting the input size to 25 × 25 × 25 can obtain a better segmentation effect. When the number of input voxels is about 3 times of the receptive field, our proposed network model can learn efficient features to improve the segmentation level.

### 3.4. Evaluate the Impact of Upsampling Strategy

The feature pyramid has multiple hierarchical structures. To make the subsequent feature fusion smoothly, it is necessary to use upsampling to keep the lower-level feature map and the adjacent upper-level feature map in the same dimension. This section uses two upsampling strategies to construct different networks and compares training and testing to evaluate the impact of these two strategies on the final segmentation effect. The data represents the average value of each index evaluated in the relevant segmentation task.

The experimental results show that the model trained using 3D deconvolution as an upsampling strategy has a better segmentation effect than the linear interpolation method. Compared with the BLInt strategy, its DSC value has been improved by 6, 4, and 4 percentage points in the segmentation evaluation of WT, TC, and EC, respectively, and the two indicators of PPV and sensitivity have also been significantly improved. First, the parameters of the 3D deconvolution filter can be learned during the network optimizing process. The weight parameters of the filter can be adaptively adjusted to appropriate values to facilitate the optimization of the objective function. Secondly, the network's use of bilinear interpolation upsampling strategy will introduce redundant information, which will affect the final segmentation effect. Therefore, DeConv is a more suitable upsampling strategy for the feature pyramid structure proposed in this chapter which is shown in Figure 5.

RETRACTED

### 3.5. Evaluate the Postprocessing Step

We evaluate CRF's effectiveness in this network for postprocessing brain tumor segmentation. Specifically, a single complete segmentation probability map is reinput to the postprocessing module for refining to obtain a structured voxel-level optimization.  Table 3 and Figure 6 show the average results of the removal/adding postprocessing method evaluated on the BraTS 2013 test set. The results show the postprocessing module can improve the segmentation performance.

## 4. Conclusion

Brain tumor is the brain disease with the highest mortality and prevalence rate. The precise segmentation of brain tumor and their intratumoral structure are important not only for treatment planning but also for follow-up evaluation. However, manual segmentation is extremely time-consuming, so we propose a simple but effective method for MRI brain tumor segmentation in this article. This paper proposes a brain tumor segmentation neural network based on a 3D hollow convolution feature pyramid. The traditional fully connected convolutional neural network has the disadvantages of too large parameter amount, fixed input size, and limited multiscale feature learning ability. A new network model is proposed to improve the accuracy of convolutional neural network segmentation of brain tumor regions and control the parameter space scale of the network model. The model first uses a convolutional layer composed of a series of 3D convolution filters to construct a backbone network for feature learning of input 3D MRI image blocks. Replace the fully connected layer with a 1 × 1 × 1 convolutional layer to make it a fully convolutional network. Then, a pyramid structure constructed by a 3D convolutional layer is designed to extract and fuse features of tumor lesions and context information of different scales and then classify the fused feature maps at the voxel level to obtain the segmentation results. Finally, a conditional random field is used to postprocess the segmentation results for structured refinement. The sensitivity of the important modules of the comparison network is analyzed through the design of many appropriate ablation experiments. The experimental results show that the algorithm in this paper can improve the segmentation performance of the algorithm on the basis of saving resources and time; compared with other algorithms, it is better in different lesion tissue regions and edge segmentation. The results confirm that the proposed network can better solve the problems mentioned above faced by the traditional fully connected convolutional neural network.

## Figures and Tables

**Figure 1:** Network structure: 3D atrous convolutional neural network, multiple feature learning, and conditional random field.

RETRACTED

**Figure 2:** Comparison with other methods: the mainstream methods include Hammoude measure (HM), multimodal magnetic resonance (MMR), fully automatic (FA), automatic brain tissue (ABT), and stereotactic brachytherapy (SBT).

**Figure 3:** Evaluate the effectiveness of atrous convolution. StdNet represents a standard convolutional neural network with a pooling layer. AConvNet.2 is the second layer of the backbone network. AConvNet.3 is the third layer of the backbone network. AConvNet.4 is the fourth layer of the backbone network.

**Figure 4:** Evaluate the impact of input size. Receptive field: 17 × 17 × 17, 25 × 25 × 25, and 37 × 37 × 37.

**Figure 5:** Evaluate the impact of upsampling strategy: BLInt and DeConv strategy.

**Figure 6:** Evaluate the effectiveness of the postprocessing step. The average results of the removal/adding postprocessing method were evaluated on the BraTS 2013 test set.

**Table 1:** The used datasets.

Dataset	Training	Testing
BraTS2013	30	35

**Table 2:** The experimental environment.

Item	Type
CPU	Intel Core i7-8700K
GPU	NVIDIA GeForce RTX 3080ti
Operating system	Ubuntu 20.04
Deep learning framework	PyTorch 1.7

**Table 3:** Evaluate the effectiveness of the postprocessing step.

3D-CRF	DSC		
	WT	TC	EC
No	0.95	0.83	0.77
Yes	0.96	0.83	0.78

## Data Availability

The datasets used and analyzed during the current study are available from the corresponding author upon reasonable request.
